# Potential of antiviral peptide-based SARS-CoV-2 inactivators to combat COVID-19

**DOI:** 10.1371/journal.pone.0268919

**Published:** 2022-06-03

**Authors:** Arun Bahadur Gurung, Mohammad Ajmal Ali, Joongku Lee, Mohamed El-Zaidy, Reem M. Aljowaie, Saeedah M. Almutairi

**Affiliations:** 1 Department of Basic Sciences and Social Sciences, North-Eastern Hill University, Shillong, Meghalaya, India; 2 Department of Botany and Microbiology, College of Science, King Saud University, Riyadh, Saudi Arabia; 3 Department of Environment and Forest Resources, Chungnam National University, Daejeon, Republic of Korea; Ghazi University, PAKISTAN

## Abstract

The appearance of new variants of severe acute respiratory syndrome coronavirus 2 (SARS-CoV-2) and the lack of effective antiviral therapeutics for coronavirus disease 2019 (COVID-19), a highly infectious disease caused by the virus, demands the search for alternative therapies. Most antiviral drugs known are passive defenders which must enter the cell to execute their function and suffer from concerns such as permeability and effectiveness, therefore in this current study, we aim to identify peptide inactivators that can act without entering the cells. SARS-CoV-2 spike protein is an essential protein that plays a major role in binding to the host receptor angiotensin-converting enzyme 2 and mediates the viral cell membrane fusion process. SARS vaccines and treatments have also been developed with the spike protein as a target. The virtual screening experiment revealed antiviral peptides which were found to be non-allergen, non-toxic and possess good water solubility. U-1, GST-removed-HR2 and HR2-18 exhibit binding energies of -47.8 kcal/mol, -43.01 kcal/mol, and -40.46 kcal/mol, respectively. The complexes between these peptides and spike protein were stabilized through hydrogen bonds as well as hydrophobic interactions. The stability of the top-ranked peptide with the drug-receptor is evidenced by 50-ns molecular dynamics (MD) simulations. The binding of U-1 induces conformational changes in the spike protein with alterations in its geometric properties such as increased flexibility, decreased compactness, the increased surface area exposed to solvent molecules, and an increase in the number of total hydrogen bonds leading to its probable inactivation. Thus, the identified antiviral peptides can be used as anti-SARS-CoV-2 candidates, inactivating the virus’s spike proteins and preventing it from infecting host cells.

## 1. Introduction

The coronavirus disease 2019 (COVID-19) is caused by the severe acute respiratory syndrome coronavirus 2 (SARS-CoV-2) virus, which became a worldwide pandemic in 2020 [1]. SARS-CoV-2 is a single-stranded, enveloped, positive-sense RNA virus belonging to the Betacoronavirus genus [2]. The genus comprises human coronavirus (HCoV)-OC43, HCoV-HKU1, Middle East respiratory syndrome coronavirus (MERS-CoV) and additionally SARS-CoV which was responsible for the 2002–2004 SARS pandemic and has 79 percent nucleotide sequence similarity with SARS-CoV-2 [1]. The SARS-CoV-2 has 14 open reading frames (ORFs), two-thirds of which encode the replicase complex’s 16 nonstructural proteins (nsp 1–16) [3, 4]. Spike mediates SARS-CoV entry into host cells, while the remaining one-third encodes nine accessory proteins (ORF) and four structural proteins: spike (S), envelope (E), membrane (M), and nucleocapsid (N) [5]. Spike comprises a receptor-binding domain (RBD) that mediates direct contact with a cellular receptor, angiotensin-converting enzyme 2 (ACE2), as well as an S1/S2 polybasic cleavage site that is proteolytically cleaved by cellular cathepsin L and the transmembrane protease serine 2 (TMPRSS2) [6–8]. Cathepsin L activates SARS-CoV-2 Spike in endosomes and can compensate for entry into cells lacking TMPRSS2 [8]. ORF1a and ORF1b are translated into viral replicase proteins once the genome is released into the host cytosol, which is then cleaved into individual nsps (through the host and viral proteases: PL^pro^), forming the RNA-dependent RNA polymerase (nsp12 generated from ORF1b) [5]. The replicase components rearrange the endoplasmic reticulum (ER) into double-membrane vesicles (DMVs), which facilitate viral replication of genomic and subgenomic RNAs (sgRNA). The latter is translated into accessory and viral structural proteins, which aid virus particle formation [9, 10].

There are currently no viable antiviral drugs or vaccines available to combat COVID-19. The majority of the antiviral drugs are referred to as "passive defenders" because they must enter virus-infected cells to prevent viral reproduction without interfering with the normal function of intracellular proteins. Passive defenders have a relatively poor utilization rate since the majority of a drug that remains outside infected cells does not engage in viral infection inhibition. Some antiviral drugs in contrast to "passive defenders," act as "gatekeepers" to battle viruses outside cells [11]. The "gatekeepers" can be divided into three categories: a) attachment inhibitors that prevent virions from attaching to target cells by blocking the binding of viral envelope glycoproteins to cellular receptors [12] (b) receptor antagonists that bind to the cell surface receptor to prevent virions from attaching to the receptor [13] c) fusion inhibitors that prevent viral and target cell membranes from fusing [14]. Attachment inhibitors, in general, have some virus inactivation properties, owing to their capacity to block the receptor-binding site on viral envelope glycoproteins [15, 16]. Virus inactivators work in a variety of ways: they can bind to and block the receptor-binding site on viral envelope glycoproteins [17], or they can cause virions to lose their ability to enter the host cell by changing the conformation of viral envelope glycoproteins [15]. Other inactivators may bind to the envelope glycoproteins stem or the viral lipid membrane, disrupting the viral envelope’s integrity or causing viral genetic contents to be released [18]. They should have a greater utilization rate than current antiviral drugs since they can actively assault and then inactivate cell-free virions everywhere in the bloodstream [11]. They should be significantly safer for *in vivo* human use than chemical-based virus inactivators which can lyse lipid membranes of viruses and cells in a non-specific manner [19].

In this present work, we have screened various antiviral peptide inhibitors to target SARS-CoV-2 spike protein using molecular docking and dynamics approaches. We anticipate that the leads identified in the study can be used as potential SARS-CoV-2 inactivators.

## 2. Materials and methods

### 2.1. Retrieval of antiviral peptide sequences

The amino acid sequences of 49 antiviral peptides with inhibitory activities against the herpes simplex virus type 1 and 2 (HSV-1 and HSV-2), MERS-CoV, SARS-CoV, human immunodeficiency virus type 1 (HIV-1), Dengue virus, Zikavirus were obtained through a literature search [11, 20]. These antiviral peptides work by one of three mechanisms: a) membrane fusion inhibition b) virus attachment inhibition, or c) virus inactivation.

### 2.2. Physicochemical property analysis of peptides

Various physicochemical properties of the peptides such as molecular weight, extinction coefficient, pI, net charge, solubility in water, toxin and allergenicity prediction using PepCalc.com-Peptide calculator (https://pepcalc.com/), ToxinPred (http://crdd.osdd.net/raghava/toxinpred/) [21] and AllerTOP v. 2.0 (https://www.ddg-pharmfac.net/AllerTOP/method.html) programs.

### 2.3. Retrieval and preparation of target enzyme

The atomic coordinates of the target enzyme spike RBD were obtained from the protein data bank (PDB) using accession ID 6M0J. The X-ray crystal structure has been resolved at a resolution of 2.45 Å containing SARS-CoV-2 spike receptor-binding domain in complex with ACE2 [22]. The heteroatoms, including ions, co-crystallized ligand, water molecules and, the ACE2 receptor were removed from the target protein.

### 2.4. Protein-peptide docking

Using the blind flexible docking approach, the HPEPDOCK web server (http://huanglab.phys.hust.edu.cn/hpepdock/) is utilised to execute blind molecular docking for peptides of various lengths into the solved structure of the SARS-CoV-2 spike receptor-binding domain (PDB ID: 6M0J). HPEPDOCK is a web-based software that uses a hierarchical algorithm to blindly dock peptides into proteins. The peptide flexibility is considered by HPEPDOCK using an ensemble of peptide conformations generated by the MODPEP program. In comparison to the well-known HADDOCK with a success rate of 45.2 percent for peptide-protein docking protocol, HPEPDOCK has a success rate of 72.6 percent for the top ten conformations. As a result, HPEPDOCK is more precise and computationally efficient [23]. To aid in the analysis of binding structures, the molecular mechanics generalized Born surface area (MM/GBSA) program of the HawkDock server [24] is used to predict the binding free energy of a protein-protein complex. The hydrogen bonds and hydrophobic interactions between the peptides and the target receptor were investigated using the DIMPLOT program of LigPlot^+^ v.1.4.5 [25].

### 2.5. MD Simulation studies

GROningen MAchine for Chemical Simulations (GROMACS) 2019.2 software package [26] with the GROMOS96 43a1 force field was used to perform simulations of the unbound SARS-CoV-2 spike and spike docked complex. Using a three-point model for water termed simple point charge (SPC216), the systems were subjected to solvation in a water-filled 3-D cube with 1 spacing. A leap-frog temporal integration technique was used for the integration of Newton’s equations of motion. The systems were neutralised, and the quantity of energy used was calculated. The systems were equilibrated for 300 ps in the NVT ensemble (Number of particles, Volume, and Temperature) and another 300 ps in the NPT ensemble (Number of particles, Volume, and Temperature) (Number of particles, Pressure and Temperature). The systems were subjected to a production MD run in an NPT ensemble for 50 ns after heating and equilibration. The Xmgrace plotting tools were used to generate the graphs.

## 3. Results

A total of forty-nine antiviral peptides were selected for the study which includes peptides against HSV-1 and 2, ZIKV, DENV, SARS-CoV-1, CoV-NL63, 229E-CoV and MERS-CoV (Table 1). The physicochemical properties such as the number of residues, molecular weight (MW), extinction coefficient, isoelectric point (pI), net charge, estimated solubility in water, toxin prediction and allergenicity were calculated for each peptide (Table 2). The peptides which displayed poor water solubility, toxin-like and allergic were discarded and the finally 14 peptides were selected for protein-peptide docking studies (Table 3). The MM/PBSA binding energy of the protein-peptide complexes is enumerated in Table 4. The best three docked peptides were U-1, HR2-18 and GST-removed-HR2 which were ranked according to the binding energy. U-1 binds to spike protein with a binding energy of -47.8 kcal/mol and the molecular interactions are mediated through six hydrogen bonds with residues Arg346, Lys444, Asn450, Glu484 and Gln493 and hydrophobic interactions with Ser349, Gly446, Tyr449, Tyr489, Phe490, Leu492 and Ser494 (Fig 1A). The second best peptide GST-removed-HR2 binds to spike protein with a binding energy of -43.01 kcal/mol and the molecular interactions are mediated through two hydrogen bonds residues Thr500 and Tyr505 and hydrophobic interactions with Lys417, Arg403, Val445, Gly446, Tyr453, Leu455, Phe456, Ala475, Tyr489, Gln493, Gly496, Gln498 and Asn501 (Fig 1B). The third best peptide HR2-18 binds to spike protein with a binding energy of -40.46 kcal/mol and the molecular interactions are mediated through four hydrogen bonds with residues Tyr453, Gln474 and Thr500 and hydrophobic interactions with Arg403, Lys417, Tyr421, Leu455, Phe456, Arg457, Tyr473, Ala475, Ser477, Gly496, Asn501 and Tyr505 (Fig 1C).

**Fig 1:** Binding poses and molecular interactions of the top-ranked peptides with spike protein (A) U-1 (B) GST-removed-HR2 (C) HR2-18. The green dashed line indicates the hydrogen bonds with distances labelled. The red and pink semi-arcs correspond to hydrophobic interacting residues of spike protein and peptide molecules respectively.

**Table 1:** List of antiviral peptides selected for *in silico* studies.

Name	Sequence	Target
gB94	KTTSSIEFARLQFTY	HSV-1
gB122	GHRRYFTFGGGYVYF	HSV-1 and 2
U-1	HRDDHETDMELKPANAATRT	HSV-1 and 2
U-2	CIGKDARDAMDRIFARRYNA	HSV-1 and 2
CB-1	QATRSETPVEVLAQQTHG	HSV-1 and 2
CB-2	PEASHRCGGQSANVEPRIL	HSV-1 and 2
Z2	MAVLGDTAWDFGSVGGALNSLGKGIHQIFGAAF	ZIKV lipid membrane
DN59	MAILDDTAWDFGSLGGVFTSIGKALHQVFGAIY	DENV lipid membrane
Urumin	IPLRGAFINGRWDSQCHRFSNGAIACA	H1 HA conserved stem
Triazole KR13	RINNIPWSEAMM	gp120 CD4bs +CoRbs
P4	EEQAKTFLDKFNHEAEDLFYQSS	SARS-CoV-1
P5	EEQAKTFLDKFNHEAEDLFYQSSLA	SARS-CoV-1
SBP1	IEEQAKTFLDKFNHEAEDLFYQS	SARS-CoV-1
RBD-11b	YKYRYL	SARS-CoV-1,CoV-NL63
SP-4	GFLYVYKGYQPI	SARS-CoV-1
SP-8	FYTTTGIGYQPY	SARS-CoV-1
SP-10	STSQKSIVAYTM	SARS-CoV-1
S471-503	ALNCYWPLNDYGFTTTGIGYQPYRVVVLSFEL	SARS-CoV-1
229E-HR2P	VVEQYNQTILNLTSEISTLENKSAELNYTVQKLQTLIDNINSTLVDLKWL	229E-CoV
P1	LTQINTTLLDLTYEMLSLQQVVKALNESYIDLKEL	MERS-CoV
HR2P	SLTQINTTLLDLTYEMLSLQQVVKALNESYIDLKEL	MERS-CoV
CP-1	GINASVVNIQKEIDRLNEVAKNLNESLIDLQELGKYE	SARS-CoV-1
HR1-1	NGIGVTQNVLYENQKQIANQFNKAISQIQESLTTTSTA	SARS-CoV-1
HR2-18	IQKEIDRLNEVAKNLNESLIDLQELGK	SARS-CoV-1
HR1-a	YENQKQIANQFNKAISQIQESLTTTSTA	SARS-CoV-1
GST-removed-HR2	DVDLGDISGINASVVNIQKEIDRLNEVAKNLNESLIDLQELGKYEQYI	SARS-CoV-1
HR2	ISGINASVVNIQKE IDRLNEVAKNLNESLIDLQEL	SARS-CoV-1
SARSWW-III	GYHLMSFPQAAPHGVVFLHVTW	SARS-CoV-1
SARSWW-IV	GVFVFNGTSWFITQRNFFS	SARS-CoV-1
SARSWW-V	AACEVAKNLNESLIDLQELGKYEQYIKW	SARS-CoV-1
SARSWW-I	MWKTPTLKYFGGFNFSQIL	SARS-CoV-1
SARSWW-II	ATAGWTFGAGAALQIPFAMQMAY	SARS-CoV-1
Anti-gp120	DGGNSNNESEIFRPGGGDMRDN	HIV-1/gp120
Anti-CCR5	YQVSSPIYDINYYTSEPCQKINVKQIAA	Co-receptor CCR5
PIE12-trimer	HPXXCDYPEWQWLCXXELGK	HIV gp41 N-trimer pocket
PAW	GTKWLTEWIPLTAEAEC	HIV-1 RT
E1P47	WILEYLWKVPFDFWRGV	HIV-1 Fusion Peptide
p7	KETWETWWTE	Dimerization of RT
Vpr 57–71	VEAIIRILQQLLFIH	HIV-1 IN & RT
Vpr 61–75	IRILQQLLFIHFRIG	HIV-1 IN & RT
Vif peptide	LITPKKIKPPLPSVT	HIV-1 Vif
p27	PQITLRKKRRQRRRPPQVSFNFCTLNF	WT & PI resistant HIV-1 protease
N46	QKQIANQFNKAISQIQESLTTTSTALGKLQDVVNQNAQALNTLVKQ	SARS-CoV
K12	GGASCCLYCRCH	SARS-CoV
P15	KLPDDFMGCV	SARS-CoV
M1-31	MADNGTITVEELKQLLEQWNLVIGFLFLAWI	SARS-CoV
M132-161	LMESELVIGAVIIRGHLRMAGHPLGRCDIK	SARS-CoV
S5	LPDPLKPTKRSFIEDLLFNKVTLADAGFMKQYG	SARS-CoV
S6	ASANLAATKMSECVLGQSKRVDFCGKGYH	SARS-CoV

**Table 2:** Physiochemical properties of the antiviral peptides with an asterisk indicating peptides that passed the solubility and *in silico* toxicity tests.

Peptide ID	Sequence	No. of residues	MW^a^ (g/mol)	Extinction coefficient (M-1cm-1)	pI	Net Charge at pH 7.0	Estimated Solubility in Water	Toxin Prediction	Allergenicity Prediction
gB94	KTTSSIEFARLQFTY	15	1792	1280	9.55	1	Poor	Non-Toxin	Probable non-allergen
gB122	GHRRYFTFGGGYVYF	15	1827.01	3840	9.97	2.1	Poor	Non-Toxin	Probable non-allergen
U-1*	HRDDHETDMELKPANAATRT	20	2308.45	0	5.2	-1.8	Good	Non-Toxin	Probable non-allergen
U-2	CIGKDARDAMDRIFARRYNA	20	2342.67	1280	10.01	1.9	Good	Non-Toxin	Probable allergen
CB-1*	QATRSETPVEVLAQQTHG	18	1952.09	0	5.26	-0.9	Good	Non-Toxin	Probable non-allergen
CB-2	PEASHRCGGQSANVEPRIL	19	2021.22	0	7.09	0	Good	Non-Toxin	Probable allergen
Z2	MAVLGDTAWDFGSVGGALNSLGKGIHQIFGAAF	33	3308.72	5690	5.04	-0.9	Poor	Non-Toxin	Probable non-allergen
DN59	MAILDDTAWDFGSLGGVFTSIGKALHQVFGAIY	33	3501.96	6970	4.01	-1.9	Poor	Non-Toxin	Probable non-allergen
Urumin	IPLRGAFINGRWDSQCHRFSNGAIACA	27	2961.35	5690	9.05	2	Poor	Non-Toxin	Probable allergen
Triazole_KR13	RINNIPWSEAMM	12	1461.71	5690	6.58	0	Poor	Non-Toxin	Probable allergen
P4	EEQAKTFLDKFNHEAEDLFYQSS	23	2776.91	1280	4	-3.9	Good	Non-Toxin	Probable allergen
P5*	EEQAKTFLDKFNHEAEDLFYQSSLA	25	2961.15	1280	4	-3.9	Good	Non-Toxin	Probable non-allergen
SBP1*	IEEQAKTFLDKFNHEAEDLFYQS	23	2802.99	1280	4	-3.9	Good	Non-Toxin	Probable non-allergen
RBD-11b*	YKYRYL	6	905.05	3840	9.81	2	Good	Non-Toxin	Probable non-allergen
SP-4	GFLYVYKGYQPI	12	1447.67	3840	9.43	1	Poor	Non-Toxin	Probable allergen
SP-8	FYTTTGIGYQPY	12	1410.52	3840	3.37	0	Poor	Non-Toxin	Probable allergen
SP-10	STSQKSIVAYTM	12	1315.49	1280	9.5	1	Poor	Non-Toxin	Probable allergen
S471-503	ALNCYWPLNDYGFTTTGIGYQPYRVVVLSFEL	32	3701.16	10810	3.93	-1.1	Poor	Non-Toxin	Probable allergen
229E-HR2P	VVEQYNQTILNLTSEISTLENKSAELNYTVQKLQTLIDNINSTLVDLKWL	50	5752.44	8250	4.01	-3	Poor	Non-Toxin	Probable non-allergen
P1	LTQINTTLLDLTYEMLSLQQVVKALNESYIDLKEL	35	4054.66	2560	3.79	-3	Poor	Non-Toxin	Probable non-allergen
HR2P	SLTQINTTLLDLTYEMLSLQQVVKALNESYIDLKEL	36	4141.74	2560	3.79	-3	Poor	Non-Toxin	Probable non-allergen
CP-1*	GINASVVNIQKEIDRLNEVAKNLNESLIDLQELGKYE	37	4170.63	1280	4.16	-3	Good	Non-Toxin	Probable non-allergen
HR1-1	NGIGVTQNVLYENQKQIANQFNKAISQIQESLTTTSTA	38	4153.52	1280	6.58	0	Poor	Non-Toxin	Probable non-allergen
HR2-18*	IQKEIDRLNEVAKNLNESLIDLQELGK	27	3123.51	0	4.32	-2	Good	Non-Toxin	Probable non-allergen
HR1-a*	YENQKQIANQFNKAISQIQESLTTTSTA	28	3157.4	1280	6.72	0	Good	Non-Toxin	Probable non-allergen
GST-removed-HR2*	DVDLGDISGINASVVNIQKEIDRLNEVAKNLNESLIDLQELGKYEQYI	48	5389.93	2560	3.74	-6	Good	Non-Toxin	Probable non-allergen
HR2*	ISGINASVVNIQKEIDRLNEVAKNLNESLIDLQEL	35	3893.36	0	4.01	-3	Good	Non-Toxin	Probable non-allergen
SARSWW-III	GYHLMSFPQAAPHGVVFLHVTW	22	2494.87	6970	7.99	0.3	Poor	Non-Toxin	Probable non-allergen
SARSWW-IV	GVFVFNGTSWFITQRNFFS	19	2254.5	5690	10.84	1	Poor	Non-Toxin	Probable non-allergen
SARSWW-V*	AACEVAKNLNESLIDLQELGKYEQYIKW	28	3269.68	8250	4.25	-2.1	Good	Non-Toxin	Probable non-allergen
SARSWW-I	MWKTPTLKYFGGFNFSQIL	19	2278.67	6970	10.21	2	Poor	Non-Toxin	Probable allergen
SARSWW-II	ATAGWTFGAGAALQIPFAMQMAY	23	2374.74	6970	3.66	0	Poor	Non-Toxin	Probable non-allergen
Anti-gp120*	DGGNSNNESEIFRPGGGDMRDN	22	2338.34	0	3.7	-3	Good	Non-Toxin	Probable non-allergen
Anti-CCR5	YQVSSPIYDINYYTSEPCQKINVKQIAA	28	3236.61	5120	6.18	-0.1	Poor	Non-Toxin	Probable non-allergen
PAW	GTKWLTEWIPLTAEAEC	17	1948.2	11380	3.85	-2.1	Poor	Non-Toxin	Probable non-allergen
E1P47	WILEYLWKVPFDFWRGV	17	2254.62	18350	6.77	0	Poor	Non-Toxin	Probable allergen
p7	KETWETWWTE	10	1395.47	17070	3.85	-2	Good	Non-Toxin	Probable allergen
Vpr_57–71	VEAIIRILQQLLFIH	15	1806.2	0	7.78	0.1	Poor	Non-Toxin	Probable non-allergen
Vpr_61–75	IRILQQLLFIHFRIG	15	1867.29	0	12.1	2.1	Poor	Non-Toxin	Probable non-allergen
Vif_peptide	LITPKKIKPPLPSVT	15	1632.04	0	10.99	3	Good	Non-Toxin	Probable allergen
p27*	PQITLRKKRRQRRRPPQVSFNFCTLNF	27	3387.97	0	12.42	7.9	Good	Non-Toxin	Probable non-allergen
N46	QKQIANQFNKAISQIQESLTTTSTALGKLQDVVNQNAQALNTLVKQ	46	5027.6	0	10.23	2	Poor	Non-Toxin	Probable non-allergen
K12	GGASCCLYCRCH	12	1272.51	1280	7.67	0.8	Poor	Toxin	Probable allergen
P15	KLPDDFMGCV	10	1124.33	0	3.71	-1.1	Good	Non-Toxin	Probable allergen
M1-31	MADNGTITVEELKQLLEQWNLVIGFLFLAWI	31	3606.19	11380	3.54	-3	Poor	Non-Toxin	Probable non-allergen
M132-161	LMESELVIGAVIIRGHLRMAGHPLGRCDIK	30	3285.96	0	8.84	1.1	Good	Non-Toxin	Probable allergen
S5*	LPDPLKPTKRSFIEDLLFNKVTLADAGFMKQYG	33	3754.36	1280	9.56	1	Good	Non-Toxin	Probable non-allergen
S6	ASANLAATKMSECVLGQSKRVDFCGKGYH	29	3072.51	1280	8.95	2	Good	Non-Toxin	Probable allergen

^a^: molecular weight b: isoelectric point

**Table 3:** HPEPDOCK results of selected peptides showing the top 10 binding models.

Peptides	Sequence	Rank/Docking score									
		1	2	3	4	5	6	7	8	9	10
U-1	KTTSSIEFARLQFTY	-148.022	-143.945	-137.215	-135.147	-132.278	-127.395	-126.299	-126.268	-125.321	-124.757
CB-1	QATRSETPVEVLAQQTHG	-162.029	-161.138	-150.976	-146.462	-144.182	-143.214	-142.947	-138.583	-136.829	-135.551
P5	EEQAKTFLDKFNHEAEDLFYQSSLA	-147.268	-144.513	-144.204	-144.009	-140.838	-140.555	-140.41	-140.12	-140.058	-139.771
SBP1	IEEQAKTFLDKFNHEAEDLFYQS	-151.454	-149.75	-142.833	-142.419	-142.11	-140.789	-139.511	-138.592	-133.748	-130.632
RBD-11b	YKYRYL	-172.275	-170.562	-168.745	-165.251	-164.41	-163.623	-162.915	-162.722	-162.669	-159.841
CP-1	GINASVVNIQKEIDRLNEVAKNLNESLIDLQELGKYE	-171.35	-163.28	-157.884	-148.261	-141.282	-140.124	-138.977	-136.679	-135.552	-133.275
HR2-18	IQKEIDRLNEVAKNLNESLIDLQELGK	-173.226	-156.699	-149.471	-146.806	-138.096	-135.439	-127.813	-124.845	-124.085	-124.051
HR1-a	YENQKQIANQFNKAISQIQESLTTTSTA	-198.579	-184.232	-174.547	-168.534	-158.606	-151.746	-151.034	-148.472	-148.095	-147.822
GST-removed-HR2	DVDLGDISGINASVVNIQKEIDRLNEVAKNLNESLIDLQELGKYEQYI	-165.483	-161.881	-158.404	-154.693	-153.735	-150.828	-149.001	-148.882	-146.856	-146.692
HR2	ISGINASVVNIQKEIDRLNEVAKNLNESLIDLQEL	-153.3	-148.706	-144.273	-143.856	-143.823	-142.512	-140.971	-140.6	-137.511	-137.248
SARSWW-V	AACEVAKNLNESLIDLQELGKYEQYIKW	-172.742	-172.433	-155.311	-151.787	-145.842	-144.029	-142.12	-142.095	-140.804	-139.481
Anti-gp120	DGGNSNNESEIFRPGGGDMRDN	-158.699	-147.191	-146.55	-146.345	-144.31	-143.424	-143.05	-141.893	-140.259	-137.558
p27	PQITLRKKRRQRRRPPQVSFNFCTLNF	-177.188	-173.317	-171.193	-171.059	-169.295	-168.792	-168.618	-167.563	-166.656	-163.571
S5	LPDPLKPTKRSFIEDLLFNKVTLADAGFMKQYG	-166.603	-164.69	-160.021	-145.79	-144.816	-143.619	-142.665	-142.232	-141.957	-140.539

**Table 4:** MM/PBSA binding energy analysis of spike protein-peptide complex.

Peptides	Sequence	Binding energy of complex (kcal/mol)
U-1	KTTSSIEFARLQFTY	-47.8
CB-1	QATRSETPVEVLAQQTHG	-37.21
P5	EEQAKTFLDKFNHEAEDLFYQSSLA	-28.08
SBP1	IEEQAKTFLDKFNHEAEDLFYQS	-35.62
RBD-11b	YKYRYL	-34.68
CP-1	GINASVVNIQKEIDRLNEVAKNLNESLIDLQELGKYE	-38.42
HR2-18	IQKEIDRLNEVAKNLNESLIDLQELGK	-40.46
HR1-a	YENQKQIANQFNKAISQIQESLTTTSTA	-38.99
GST-removed-HR2	DVDLGDISGINASVVNIQKEIDRLNEVAKNLNESLIDLQELGKYEQYI	-43.01
HR2	ISGINASVVNIQKEIDRLNEVAKNLNESLIDLQEL	-20.65
SARSWW-V	AACEVAKNLNESLIDLQELGKYEQYIKW	-32.74
Anti-gp120	DGGNSNNESEIFRPGGGDMRDN	-31.84
p27	PQITLRKKRRQRRRPPQVSFNFCTLNF	-22.14
S5	LPDPLKPTKRSFIEDLLFNKVTLADAGFMKQYG	-35.2

The top-ranked peptide U-1 complex with spike protein and unbound spike protein were subjected to MD simulations for 50 ns in an aqueous environment and various structural properties were derived from their trajectories (Table 5). The root-mean-square deviation (RMSD) is a measurement of the structural deviation of atomic positions and is an important parameter for evaluating the stability of protein structures. The average RMSD of Spike protein and Spike_U-1 complex was found to be 0.268143±0.042207 nm and 0.311734±0.034062 nm respectively (Table 3). The peptide binding causes an enhancement in the structural flexibility of the spike protein as evident from the RMSD plot (Fig 2). An average of the residual fluctuations in the SARS-CoV-2 spike was determined and plotted as the root-mean-square fluctuation (RMSF) to explore the local fluctuations in the target protein before and after the binding of the peptide (Fig 3). The RMSF plot revealed increased amplitudes of fluctuations after peptide binding to the receptor. The radius of gyration (Rg) is a parameter to evaluate protein stability and folding behaviour and gives an idea of the overall structural shape of a protein. The Rg of Spike protein and Spike_U-1 complex were calculated to determine their structural compactness (Fig 4). The Rg values of Spike protein and Spike_U-1 complex were 1.743737±0.029687 nm and 1.803292±0.012467 nm respectively. The complex has a higher Rg and maintains a stable equilibrium after 20 ns when compared to free spike protein. Further, the Rg plot analysis suggests that the spike protein undergoes conformational changes resulting in decreased structural compactness with the binding of the peptide. The solvent-accessible surface area (SASA) of a protein is the region of the protein that interacts directly with its surrounding water molecules. During the 50 ns MD simulation, the SASA plot for Spike protein and Spike_U-1 complex were generated (Fig 5). The average SASA values for Spike protein and Spike_U-1 complex were determined to be 98.04472±2.837382 nm^2^ and 106.8303±2.801777 nm^2^ respectively. An increase in SASA value was observed due to the conformational changes in the target protein after interaction with the peptide. The stability and overall shape of a protein are dependent on the hydrogen bond network. The average number of hydrogen bonds in Spike and U-1_spike complex were 123.99±6.897963 and 214.8142±7.892619 respectively which help to stabilize the protein-peptide complex. Hydrogen bonds formed during the simulation were computed and displayed to confirm the stability of Spike protein and Spike_U-1 complex (Fig 6).

**Fig 2:** Plot of RMSD vs time (ps) for unbound spike protein (blue) and spike_U-1 complex (red).

**Fig 3:** Plot of RMSF vs residue for unbound spike protein (blue) and spike_U-1 complex (red).

**Fig 4:** Plot of Rg vs time (ps) for unbound spike protein (blue) and spike_U-1 complex (red).

**Fig 5:** Plot of number of Total SASA vs time (ps) for unbound spike protein (blue) and spike_U-1 complex (red).

**Fig 6:** Plot of number of hydrogen bonds vs time (ps) for unbound spike protein (blue) and spike_U-1 complex (red).

**Table 5:** Geometric properties of unbound spike protein and its complex with U-1 peptide.

Parameters	Spike protein	Spike_U-1 complex
**RMSD (nm)**	0.268143±0.042207	0.311734±0.034062
**Rg (nm)**	1.743737±0.029687	1.803292±0.012467
**Total SASA (nm** ^**2**^ **)**	98.04472±2.837382	106.8303±2.801777
**Number of Hydrogen bonds**	123.99±6.897963	142.2735±7.201047

## 4. Discussion

The coronavirus disease 2019 (COVID-19) became a global pandemic in 2020 and currently, there are no effective antiviral drugs or vaccines against it. Further, the emergence of different variants of SARS-CoV-2 such as delta and omicron has posed a serious threat to global health around the world [27, 28]. In this present work, we have screened peptides as inhibitors of SARS-CoV-2 by targeting the spike protein RBD using molecular docking and dynamics approaches. Virtual screening of 49 antiviral peptides yield 14 peptides which were found to be non-allergic, non-toxic, good water solubility. These selected peptides were investigated for their binding potential to spike protein, a surface glycoprotein that is a target for the majority of current vaccines and which is essential for recognising and binding to the host cell surface receptor. Three peptides-U-1, GST-removed-HR2 and HR2-18 were identified which show high binding affinity to SARS-CoV-2 spike protein. U-1 is an antiviral peptide (AVP) derived from the continuous residue stretches (CRSs) located at the surface of glycoprotein B (gB) (residues 224–243, HRDDHETDMELKPANAATRT) which has high *in vitro* virucidal and antiviral activities against both herpes simplex viruses type 1 (HSV-1) and type 2 (HSV-2) [29]. GST-removed-HR2 is a recombinant protein derived from the heptad repeat 2 (HR2) region (residues 1145–1192, DVDLGDISGINASVVNIQKEIDRLNEVAKNLNESLIDLQELGKYEQYI) which inhibits viral entry in Vero E3-luciferase assay (EC_50_ = 2.15 μM) and functions as SARS-CoV entry inhibitors [30]. HR2-18 is a potent entry inhibitor of SARS-CoV (EC_50_ = 1.19 μM) in 293T-luciferase assay derived from HR2 regions in the S2 protein (residues 1161–1187, IQKEIDRLNEVAKNLNESLIDLQELGK) which can serve as a functional probe to unravel the fusion mechanism of SARS-CoV [31]. The stability of the best lead peptide U-1 with the spike protein was assessed in terms of MD derived geometric properties such as RMSD, RMSF, SASA, number of hydrogen bonds. The binding of U-1 to spike protein causes conformational changes such as an increase in the flexibility of the protein, a decrease in the compactness of the protein, an increase in the surface area exposed to solvent molecules and an increase in the number of total hydrogen bonds. We anticipate that the leads identified in the study can be used as potential inhibitors of the SARS-CoV-2 spike by acting as virus inactivators which will prevent the entry of the virus into the host cells and subsequently halt the virus multiplications. Such peptide inactivators have added advantages of being able to act on the virus even when outside the cells, enhanced efficiency and eliminating the requirement for these peptides to penetrate the cells.

## 5. Conclusion

The lack of effective therapeutic drugs against SARS-CoV-2 infections and the continued rise in the fatality rate warrant the identification of novel therapeutics. SARS-CoV-2 spike is an important protein for receptor recognition and cell membrane fusion. In our study, we have explored the possibilities of major antiviral peptides to inhibit the interaction between Spike and ACE2 using a combined approach of molecular docking and dynamics simulation. We identified three antiviral peptides-U-1, GST-removed-HR2 and HR2-18 which exhibit high binding affinities to the spike protein. Wet-lab experimentations are required to validate our findings before they may proceed into the development of an anti-SARS-CoV-2 therapeutic candidate.
